# Gene Characteristics and Prognostic Values of m^6^A RNA Methylation Regulators in Nonsmall Cell Lung Cancer

**DOI:** 10.1155/2021/2257066

**Published:** 2021-07-29

**Authors:** Na Li, Xiaojuan Chen, Yanhong Liu, Tieming Zhou, Wei Li

**Affiliations:** ^1^Department of Pathology, The Second Affiliated Hospital of Hunan University of Chinese Medicine, Changsha, China; ^2^Department of Clinical Laboratory, Maternal and Child Care Hospital, Changsha, Hunan, China; ^3^Department of Geriatrics, Clinical Laboratory, Xiangya Hospital of Central South University, Changsha, China

## Abstract

**Background:**

N^6^-methyladenosine (m^6^A) is the most common internal modiﬁcation present in mRNAs and long noncoding RNAs (lncRNAs), associated with tumorigenesis and cancer progression. However, little is known about the roles of m^6^A and its regulatory genes in nonsmall cell lung cancer (NSCLC). Here, we systematically explored the roles and prognostic significance of m^6^A-associated regulatory genes in NSCLC.

**Methods:**

The copy number variation (CNV), mutation, mRNA expression data, and corresponding clinical pathology information of 1057 NSCLC patients were downloaded from the cancer genome atlas (TCGA) database. The gain and loss levels of CNVs were determined by utilizing segmentation analysis and GISTIC algorithm. The GSEA was conducted to explore the functions related to different levels of m^6^A regulatory genes. Logrank test was utilized to assess the prognostic significance of m^6^A-related gene's CNV.

**Results:**

The genetic alterations of ten m^6^A-associated regulators were identified in 102 independent NSCLC samples and significantly related to advanced tumor stage. Deletions or shallow deletions corresponded to lower mRNA expression while copy number gains or amplifications were related to increased mRNA expression of m^6^A regulatory genes. Survival analysis showed the patients with copy number loss of *FTO* with worse disease-free survival (DFS) or overall survival (OS). Besides, copy number loss of *YTHDC2* was also with poor OS for NSCLC patients. Moreover, high *FTO* expression was significantly associated with oxidative phosphorylation, translation, and metabolism of mRNA.

**Conclusion:**

Our findings provide novel insight for better understanding of the roles of m^6^A regulators and RNA epigenetic modification in the pathogenesis of NSCLC.

## 1. Introduction

Lung cancer is one of the most prevalent malignant tumors and also the most lethal cancer with an approximate 5-year survival rate of 16% all over the world [1]. The latest cancer statistic data indicate that there will be 19,300,000 new tumor patients and more than 10,000,000 deaths in 2020 [1, 2]. Nonsmall cell lung cancer (NSCLC) is the most prevalent type of lung tumor which accounts for 80% of all cases. In the past decades, a series of therapeutics including chemotherapy, surgery, radiotherapy, and immunotherapy were applied to lung tumor patients; however, the prognosis of patients is still unfavorable and is especially poor in advanced NSCLC [3]. NSCLC has become a serious health problem worldwide. Hence, to further explore the molecular pathogenesis underlying NSCLC to develop effective diagnostics and therapies is urgently needed.

The genetic and epigenetic alterations of nucleotides were involved in various regular bioprocesses such as regulation of gene expression, variable splicing, and protein translation, which play essential roles in the occurrence and progression of various diseases [4–6]. RNAs nucleotides modification is a common epigenetic alteration and more than 100 chemically modified nucleotides in different RNAs have been identified [7, 8]. Among these, methylation of N^6^-methyladenosine (m^6^A) is the most prevalent internal form of messenger RNAs (mRNAs) and long noncoding RNAs (lncRNAs) modification in eukaryotes [9]. Previous studies have shown that m^6^A modification is present in more than 7,600 mRNAs and in over 300 noncoding RNAs [10]. It is known as m^6^A modification closely related to RNA splicing, localization, stability, export, RNA-protein interactions, alternative polyadenylation, and translation [11–13]. The cellular m^6^A methylation is mediated by a group of regulatory enzymes including “writers” Wilms' tumor 1-associated protein (WTAP), methyltransferase-like 3 (METTL3) and METTL14, “erasers” fat mass and obesity-associated protein (*FTO*) and alkB homolog 5 (ALKBH5), and “readers” YTH domain containing 1 (YTHDC1/2) and YTH N^6^-methyladenosine RNA binding protein 1/2/3 (YTHDF1/2/3) [14–16]. Generally, m^6^A methylation is increased by writers, erased by *FTO* or ALKBH5, and deciphered by YTHDF1/2/3 or YTHDC1/2.

In recent years, growing evidences indicated that m^6^A dysregulation plays critical roles in tumorigenesis and cancer progression through diverse molecular mechanisms [14–18]. Meanwhile, the expression level of m^6^A-related regulatory proteins has been shown to be critically involved in tumorigenesis [19–21]. Knockout of m^6^A methyltransferase can regulate cancer occurrence by affecting the activity of p53 signaling pathway [22]. More recently, downregulation of *FTO* reduced lung cancer cell proliferation and invasion and promoted cell apoptosis [23, 24]. Another study also revealed that *METTL14* by regulating its mRNA targets promotes leukemogenesis through mRNA m^6^A modification [25]. All these results show that m^6^A modiﬁcation factors play essential roles in the occurrence of a variety of cancers. However, the connection between m^6^A-related regulatory factors and NSCLC remained not very clear. In the present work, we systematically explored the expression pattern of m^6^A regulators in NSCLC based on the data from TCGA database. We also analyzed the association between m^6^A-related genetic alterations and clinical features including age, sex, pathological stage, disease-free survival (DFS), and overall survival (OS).

## 2. Materials and Methods

### 2.1. Acquisition of NSCLC Data

The CNV, mutation, mRNA expression information, and corresponding clinicopathological information of 1057 NSCLC patients were obtained from the TCGA database (GDC data portal) (https://cancergenome.nih.gov/).

### 2.2. Data Preprocessing and Copy Number Variations Identifying

The gain and loss levels of copy number variations (CNVs) were determined by utilizing segmentation analysis and GISTIC algorithm.

The NSCLC samples were grouped into two classes: without CNVs and mutation of ten m^6^A regulators and with CNVs and/or mutation. The expression of mRNA in each CNV groups was calculated using R package “DESeq2.”

### 2.3. Gene Set Enrichment Analysis (GSEA)

The GSEA was implemented to explore the functions related to different levels of m^6^A regulatory genes.

The JAVA program with MSigDB v6.1 was used to execute GSEA. All samples were sorted into low- and high-*FTO* level groups. Then, significant enrichment of gene sets was calculated with a false discovery rate (FDR) value less than 0.25 and a normalized *P* value less than 0.05.

### 2.4. Survival Analysis

All NSCLC samples were grouped by with or without deletion/gain of each m^6^A regulator gene and then a survival analysis was conducted by utilizing R packages “survival” (https://cran.r-project.org/web/packages/survival/index.html) and R package “survminer” (https://cran.r-project.org/web/packages/survminer/index.html). The prognosis value of the CNV of m^6^A regulatory gene was assessed by logrank test. Moreover, the Kaplan–Meier plotter (https://kmplot.com/analysis/) was used to analyze the prognosis value of each m^6^A regulator.

### 2.5. Statistical Analysis

All data were processed by utilizing R (4.0). The relationship between the CNV of m^6^A regulators and clinical-pathological features was investigated with chi-square test or Kruskal–Wallis rank sum test. All *P* values less than 0.05 were treated to be statistically significant.

## 3. Results

### 3.1. Mutations and CNV Events of m^6^A Regulators in NSCLC Samples

In total, 1057 NSCLC specimens with sequencing data were included in the present research. Among these, the genetic alterations of m^6^A moderators were identified in 102 independent samples (Figure 1). In detail, the m^6^A “reader” genes *YTHDF3* (8.8%, 93/1057), *YTHDF1* (7.85%, 83/1057), and *YTHDC2* (5.58%, 59/1057) are the top three genes in the CNVs frequency (Table 1, Figure 2(a)). Moreover, the CNVs of NSCLC-driven genes *EGFR*, *KRAS,* and *TP53* were assessed and the results were 13.43%, 10.69%, and 6.53% (Table 1, Figure 2(a)), respectively. Subsequently, we counted all CNV patterns in NSCLC samples and found that the copy number loss events are the most of all CNVs (264/495) (Table 1, Figure 2(b)). The shallow deletions of *YTHDC2* are the most frequent copy number loss of these ten m^6^A regulators, while the gain of *YTHDF3* DNA copy number is the most common change in the CNVs of ten m^6^A regulatory genes (Table 1, Figure 2), suggesting a key significance of m^6^A reader genes in RNA m^6^A methylation in NSCLC patients.

### 3.2. Association between the Alterations of m^6^A Regulators and Clinical-Pathological Characteristics

To investigate the connection between genetic variations of m^6^A regulators and the clinicopathological characteristics of NSCLC patients, we implemented a correlation analysis. The results showed that genetic alterations of m^6^A-related regulators were obviously correlated to advanced tumor stage (*P* < 0.05) (Table 2). Given that *EGFR*, *TP53*, and *KRAS* play crucial roles in tumorigenesis and progression of lung cancer, we examined the connection between m^6^A-related regulators and the variations of the above three tumor-related genes. We found that the variations of m^6^A regulatory genes were obviously linked to *EGFR* and *TP53* alteration (*P* < 0.05) (Table 3). In detail, only 54 samples were missing from alterations of m^6^A regulators among the 316 patients with *EGFR* alteration and 57 samples were absent in 321 patients with *TP53* alteration (Table 3). However, variations of m^6^A regulators did not correlate significantly with *KRAS* mutation (*P* > 0.05) (Table 3).

Subsequently, we further explored whether alterations in m^6^A-related genes affect mRNA expression. The results suggested that the expression of mRNA was significantly related to different CNV types in NSCLC patients. Deletions or shallow deletions were corresponding to lower mRNA expression while copy number gains or amplifications were linked to increased mRNA expression of the ten m^6^A regulators (Figure 3).

### 3.3. Prognostic Significance of CNVs in m^6^A Regulatory Genes for NSCLC Patients

The prognostic significance of CNVs in the m^6^A regulators for DFS and OS among NSCLC patients was investigated, there was no significant correlation between patients with/without CNVs of m^6^A-related regulators and OS or DFS (Figures 4(a)-4(b)). However, further analysis showed copy number loss of *FTO* with worse DFS and OS (Figures 4(c)-4(d)). Besides, copy number loss of *YTHDC2* is also with poor OS for NSCLC patients (Figure 4(e)). Furthermore, we further found low *FTO* expression was closely related to poor OS of lung cancer patients by using Kaplan–Meier plotter (Figure 4(f)).

### 3.4. Enrichment Analysis of *FTO* Gains of Function

Given that there is close correlation between CNVs and m^6^A regulator *FTO* and NSCLC prognosis, a GSEA was executed to investigate the gene enrichment in patients with different *FTO* mRNA expression. The results showed that high *FTO* expression was significantly associated with multiple key biological processes, including oxidative phosphorylation, ribosome, translation, 3′-UTR-mediated translational regulation, metabolism of mRNA, and influenza life cycle (Figure 5), which provides new clues for understanding the pathogenesis of NSCLC.

## 4. Discussion

RNA modification is an emerging branch of epigenetics that is increasingly attracting the interest of related researchers. Currently, RNA modification is thought to be widespread in almost all forms of RNA, including mRNAs, lncRNAs, rRNAs, tRNAs, micro-RNAs, and small nucleolar RNAs [26–28]. Previous studies have shown that RNA modifications include multiple forms, such as pseudouridine, N7-methyladenosine, 2′-O-methylation, N1-methyladenosine, N6,2-O-dimethyladenosine (m^6^A), and 5-methylcytosine [29, 30]. Among them, m^6^A methylation is the most common mRNA modification form and it participates in the regulation of numerous biological processes in eukaryotes [29–31]. The cellular m^6^A status is dynamically regulated by methyltransferases, binding proteins, and demethylases. The alterations of these regulatory factors lead to dysregulation of m^6^A methylation and hence play an essential role in the progression of various diseases [31–33].

Bioinformatics analysis plays a fundamental role in disease diagnosis and pathogenesis research [34–36]. In this study, we used bioinformatics approaches to systematically identify the roles and prognostic values of m^6^A-related regulatory factors in NSCLC. A total of 1057 NSCLC samples with CNV information and clinical data from TCGA were included. Of these, 102 independent samples were identified as having the genetic variations of m^6^A-related regulators. Compared with clear cell renal cell carcinoma (ccRCC) and acute myeloid leukemia, the frequency of alterations in ten m^6^A-related genes in lung cancer is less [37, 38]. Among all CNV patterns in NSCLC, the copy number loss was the most important part of all CNV events, which was similar as the CNV patterns in ccRCC [37] and acute myeloid leukemia [38]. For all m^6^A regulators, deletions are the most important part of CNVs in “eraser” and “writer” genes, but the number of gain of CNV events in “eraser” genes is higher than those of “writer” genes, which eventually decreased the m^6^A level in NSCLC cells. Previous studies have shown that m^6^A levels were downregulated in various tumors, such as glioblastoma and breast cancer [39–41]. This may also be explained by the opposite effect on m^6^A status for“eraser” and “writer” genes.

Furthermore, we found that copy number gains or amplifications were positively correlated with mRNA levels of the 10 m^6^A-related regulators while deletions or shallow deletions were negatively related to mRNA levels, implying that alterations in CNVs affect m^6^A-related genes expression in NSCLC. Further analysis revealed that alterations of m^6^A-related regulators were positively linked to cancer stage of NSCLC. These results suggested that CNVs of m^6^A regulatory genes are involved in the regulation of tumor progression by affecting methylation modification of RNAs. A recent study found that overexpression of m^6^A methyltransferase *METTL3* facilitates tumor development through AFF4/NF-*κ*B/MYC signal pathway in bladder cancer [42]. Another study also indicated changes in the expression of m^6^A regulatory genes by regulating corresponding genes to promote breast cancer progression [41]. We also found that the changes of m^6^A modulators were significantly associated with *EGFR* and *TP53* alteration. EGFR is an important oncogene, and its mediated pathways play crucial roles in tumor occurrence and development [43–45], while *TP53* is a classic tumor suppressor gene [46]. Based on these findings, we speculate that dysregulated m^6^A status induced *EGFR* activation and *TP53* inactivation to facilitate the tumorigenesis and progress of NSCLC.

Moreover, we explored the prognostic value of m^6^A regulator alterations in NSCLC. For all ten m^6^A-related genes, only copy number loss of eraser gene *FTO* and reader gene *YTHDC2* was significantly associated with poor survival status for NSCLC patients. Besides, the results of Kaplan–Meier plotter analysis also indicate that low *FTO* expression is related to worse OS of lung cancer patients. Taking together, the present results showed that the *FTO* levels are inversely related to the survival time of patients with NSCLC. However, studies have revealed that *FTO* as an m^6^A demethylase participates in promoting the growth of lung cancer cells in vitro [23, 24]. These findings revealed that m^6^A regulatory genes are a “double-edged sword” in tumorigenesis, which could lead to not only tumor suppression but also tumor progression. Thus, restoring the balanced state of RNA methylation in tumor cells is a new anticancer strategy.

The present study displayed that m^6^A-related regulatory genes were also associated with multiple signaling pathways and biological processes of NSCLC occurrence and development. The results of the GSEA suggested that the expression of FTO was significantly related to oxidative phosphorylation, ribosome, translation, 3′-UTR-mediated translational regulation, and metabolism of mRNA. Similar to our results, a previous study reported that *FTO* expression was positively related to dextrose oxidation rates and levels of genes related to oxidative phosphorylation in skeletal muscle [47]. It has been shown that oxidative phosphorylation plays significant roles in lung cancer proliferation, invasion, metastasis, and drug resistance [48–50]. Therefore, it is likely that genetic alterations of *FTO* regulate the progression of NSCLC by affecting cellular oxidative phosphorylation levels. The specific molecular mechanism deserves to be explored through further work. In addition, several biological processes regulated by the m^6^A regulators have been identified, including RNA metabolism, translational regulation, and protein translation [23, 51], which are consistent with our GSEA results.

In conclusion, our work systematically displayed the genetic alterations, expression patterns, potential roles, and prognostic significance of m^6^A-related regulators in NSCLC and found that the alterations of m^6^A regulators are highly related to the malignant clinicopathological characteristics including survival. These results help us to find out the functions of m^6^A RNA methylation in the pathogenesis of NSCLC. However, these findings need to be validated with further clinical and molecular biology experiments.

## Figures and Tables

**Figure 1:** CNVs and mutations of top ten m^6^A regulators in NSCLC patients.

**Figure 2:** CNVs of ten m^6^A regulators in NSCLC. (a) CNV ratio of m^6^A regulators in NSCLC samples. (b) Number of gain or loss of DNA copy number of m^6^A-related regulators in NSCLC patients.

**Figure 3:** The relation between CNV types and m^6^A regulator expression.

**Figure 4:** Survival analysis of NSCLC patients with CNVs of m^6^A-related regulators. ((a)-(b)) OS and DFS for NSCLC patients who have any alteration of m^6^A-related regulators, ((c)-(d)) DFS and OS for patients with NSCLC who have different CNV types of *FTO*, (e) OS for patients with NSCLC who have different CNV types of *YTHDC2*, and (f) OS for patients with *FTO* mRNA expression levels by Kaplan–Meier plotter.

**Figure 5:** GSEA outcomes of different expression level of *FTO*. (a) Oxidative phosphorylation, (b) ribosome, (c) translation, (d) 3′-UTR-mediated translational regulation, (e) metabolism of mRNA, and (f) influenza life cycle.

**Table 1:** CNV patterns in NSCLC patients (*N* = 1057).

Gene		Diploid	Deep deletion	Shallow deletion	Copy number gain	Amplification	CNV sum	Percentage
Eraser	ALKBH5	999	0	45	11	2	58	5.49
	FTO	1004	2	30	20	1	53	5.01

Writer	METTL14	1034	1	21	1	0	23	2.18
	METTL3	1032	1	20	1	3	25	2.37
	WTAP	1004	1	39	12	1	53	5.01

Reader	YTHDF1	974	0	8	67	8	83	7.85
	YTHDF2	1027	0	24	6	0	30	2.84
	YTHDC1	1039	0	12	1	5	18	1.70
	YTHDC2	998	1	53	4	1	59	5.58
	YTHDF3	964	0	6	81	6	93	8.80

Others	EGFR	915	4	12	82	44	142	13.43
	KRAS	944	4	9	72	28	113	10.69
	TP53	988	4	55	8	2	69	6.53

**Table 2:** Clinical features of patients with NSCLC who are with or without genetic alterations of m^6^A regulators.

Parameters		With mutation and/or CNVs	Without mutation and/or CNVs	*P* value
Age	≤60	90	176	0.217
	>60	223	524	

Gender	Female	123	283	0.787
	Male	190	417	

Primary diagnosis	Acinar cell carcinoma	6	16	0.07
	Adenocarcinoma, NOS	102	210	
	Adenocarcinoma with mixed subtypes	37	71	
	Basaloid squamous cell carcinoma	5	9	
	Bronchiolo-alveolar carcinoma, mucinous	2	3	
	Bronchiolo-alveolar adenocarcinoma, NOS	1	2	
	Bronchiolo-alveolar carcinoma, nonmucinous	6	12	
	Clear cell adenocarcinoma, NOS	1	1	
	Micropapillary carcinoma, NOS	0	3	
	Mucinous adenocarcinoma	1	12	
	Papillary adenocarcinoma, NOS	6	16	
	Papillary squamous cell carcinoma	1	3	
	Signet ring cell carcinoma	0	1	
	Solid carcinoma, NOS	2	4	
	Squamous cell carcinoma, keratinizing, NOS	3	9	
	Squamous cell carcinoma, small cell, nonkeratinizing	1	3	
	Squamous cell carcinoma, NOS	139	325	

Tumor stage	Not reported	3	8	**0.001** ^*∗*^
	Stage I-II	242	559	
	Stage III-IV	68	133	

Tissue or organ of origin	Lower lobe, lung	99	251	0.137
	Lung, NOS	14	37	
	Main bronchus	4	5	
	Middle lobe, lung	14	23	
	Overlapping lesion of lung	6	5	
	Upper lobe, lung	176	379	

NOS, not otherwise specified.

**Table 3:** Relationship between EGFR/KRAS/TP53 and m^6^A genes.

Gene		With alteration in 10 m^6^A genes	Without alteration in 10 m^6^A genes	*χ* ^2^	*P* value
EGFR	WT	262	629	6.598	**0.010**
*n* = 1023	Alteration	54	78		

TP53	WT	264	694	96.505	**<0.001**
*n* = 1024	Alteration	57	9		

KRAS	WT	283	647	2.039	0.153
*n* = 1036	Alteration	40	66		

## Data Availability

Publicly available datasets were analyzed in this study. These data can be found at https://www.cancer.gov/.
